# The Effects of Cytokines in Adipose Stem Cell-Conditioned Medium on the Migration and Proliferation of Skin Fibroblasts *In Vitro*

This article has been retracted.

**DOI:** 10.1155/2013/578479

**Published:** 2013-12-15

**Authors:** Jiajia Zhao, Li Hu, Jiarong Liu, Niya Gong, Lili Chen

**Affiliations:** Department of Stomatology, Union Hospital, Tongji Medical College, Huazhong University of Science and Technology, Wuhan 430022, China

## Abstract

Although adipose stem cell-conditioned medium (ASC-CM) has demonstrated the effect of promoting the cutaneous wound healing, the mechanism for this response on the effector cells (e.g., dermal fibroblasts) during the process remains to be determined. In this study, we aim to investigate the types and contents of cytokines in ASC-CM and the effects of some kinds of common cytokines in ASC-CM, such as EGF, PDGF-AA, VEGF, and bFGF, on dermal fibroblasts proliferation and migration in wound healing process. Results showed that these four cytokines had high concentrations in ASC-CM. The migration of skin fibroblasts could be significantly stimulated by VEGF, bFGF, and PDGF-AA, and the proliferation could be significantly stimulated by bFGF and EGF in ASC-CM. Additionally, ASC-CM had more obvious promoting effect on fibroblasts proliferation and migration than single cytokine. These observations suggested that ASC-CM played an important role in the cutaneous injury partly by the synergistic actions of several cytokines in promoting dermal fibroblasts proliferation and migration, and ASC-CM was more adaptive than each single cytokine to be applied in promoting the wound healing.

## 1. Introduction

During the last decade, adipose-derived stem cells (ASCs) have been gaining increasing attention in tissue repair therapeutic application since they were first isolated from adipose tissues in 2001 [1–3]. ASCs are a population of multipotent mesenchymal cells, with similar characteristics to bone marrow-derived mesenchymal stem cells (BM-MSCs), which are classical cell source for tissue regeneration. Furthermore, compared with BM-MSCs, ASCs have been shown to be immunoprivileged and appear to be more genetically stable in long-term culture [4–6].

Numerous studies have indicated that ASCs may contribute to tissue injury repair or regeneration. In recent years, the mechanisms of ASCs promoting tissue wound healing caused huge attention, and the paracrine mechanism might be the most effective way for ASCs to promote wound healing; that is, they exert their effect by secreting cytokines and growth factors acting on neighboring cells to repair damaged tissues [7–9]. ASC-conditioned medium (ASC-CM) contained a great many biologically active factors secreted by ASCs, and it has the distinct advantage of being applicable via local or intravenous injection. More importantly, the contents of major cytokines in the ASC-CM can be precisely quantitated. Thus, ASC-CM has its good application prospects.

Fibroblasts, one of the dominant components of dermal structure, serve as critically important function all through the whole skin wound healing process. In the early stage of wound healing, they migrate to the traumatized region to promote the regeneration of blood vessels and granulation tissue formation via secreting some angiogenesis factors. And in the advanced trauma repair, a large number of fibroblasts mature into myofibroblasts, which are conducive to promoting wound closure [10, 11]. Therefore, the migration and proliferation of fibroblasts are the key links in wound healing process, and the elucidation of the mechanism behind the effects of ASC-CM on fibroblasts migration and proliferation would contribute to the optimization of the clinical application of ASC-CM to wound healing.

However, it is so far unknown whether there is a correlation between the ASC-CM concentration and the efficacy of ASC-CM in promoting the migration and proliferation of skin fibroblasts. Since there are very few reports on the main functional factors in ASC-CM and their action mechanism, a thorough investigation of these issues, which is the focus of this study, will contribute to a better understanding of the ASC paracrine mechanism and ultimately lead to an improved use of ASC-CM in wound healing. 

## 2. Materials and Methods

### 2.1. Isolation, Culture, and Identification of Primary Human Skin Fibroblasts

Skin fibroblasts were isolated and cultured as previously described [12]. Briefly, human foreskins were obtained aseptically from donors (16–30 years old) undergoing circumcision after obtaining their written informed consent. All the procedures were approved by the Ethics Committee of Wuhan Union Hospital. The samples were washed several times with 75% alcohol and sterile PBS (Hyclone, Thermo Scientific, USA) containing 1% antibiotic (100 U/mL penicillin/streptomycin) and were treated with 4 mg/mL dispase II (Gibco, USA) overnight at 4°C to separate epidermis and dermis [12]. The dermis was then cut into small pieces and digested with 0.1% collagenase type I (Gibco, USA) for 4 hours at 37°C to isolate fibroblasts. Cells were cultured at 37°C in 5.0% CO_2_ and medium was changed every 2-3 days. P3 cells were used for immunofluorescence staining of vimentin and cytokeratin 15 (Santa Cruz, USA).

### 2.2. Isolation, Characterization, and Multidifferentiation Assay of ASCs

Human subcutaneous adipose tissues were obtained from female patients (18–35 years old) undergoing lipoaspiration surgery after obtaining written informed consent and approval by the Ethics Committee of Wuhan Union Hospital. The procedures described by Hu et al. were utilized for this purpose [13]. Cells were cultured in specific mesenchymal stem cells culture medium (Cyagen) and P3–P7 cells were used for the present study. The surface markers CD13, CD14, CD44, CD90, CD105, and CD34 were tested by flow cytometry and analyzed by a standard Becton-Dickinson FACSAria instrument and the CellQuest Pro software (BD Biosciences). After ASCs had been diversely differentiated into multiple lines, the adipogenic lineage was detected by Oil-Red-O (Sigma) staining for lipid droplets, and the osteogenic lineage was detected by alizarin red (Sigma) staining for calcium depositions. At the same time, the expression of peroxisome proliferator-activated receptor gamma (PPAR-*γ*) was tested by RT-PCR during the adipogenesis process and runt-related transcription factor 2 (Runx2) was tested during the osteogenesis process.

### 2.3. Preparation of ASC-CM and Protein Microarray Analysis

ASCs were cultured until reaching 80% confluence. The culture medium was then replaced with serum-free DMEM/F-12, and ASCs were cultured for another 48 hours. The ASCs-conditioned medium (ASC-CM) was collected, centrifuged at 1,000 rpm for 5 minutes, and filtered through 0.22 *μ*m syringe filter. Thus, the ASC-CM contained DMEM/F-12 and any factors secreted by ASCs. ASC-CM was stored at −20°C, and 5 mL medium was used for protein array analysis with the RayBio Biotin Label-based Human Antibody Array I (Cat. No. AAH-BLM-1-2, Norcross, GA) which contains antibodies for 507 human proteins. Three ASC-CM samples (ASCs were derived from three different donors) were used to do protein microarray analysis.

### 2.4. Migration Assays

The effect of ASC-CM on cell migration was determined by transwell assay and scrape-wound healing assay. In transwell assay, 1 × 10^5^ fibroblasts were seeded into the upper chamber of the insert (transwell plates are 6.5 mm in diameter with 8 *μ*m pore filters; Corning Costar, Cambridge, MA), with 300 *μ*L of culture medium in upper chamber and 600 *μ*L medium in lower chamber. After the cells adhered, the medium in the upper chamber was changed with serum-free DMEM/F-12. To determine the respective effects and the optimal concentrations of EGF, PDGF-AA, VEGF, and bFGF in ASC-CM, the culture medium in the lower chamber was changed with (i) 50% ASC-CM, which was the optimal ASC-CM concentration for promoting fibroblasts migration in our previous study [13], with different concentrations of cytokines (EGF, PDGF-AA, VEGF, and bFGF, at 0, 1, 10, 20, 50, and 100 ng/mL, resp.), (ii) 50% ASC-CM with the neutralizing antibody of each cytokine, or (iii) serum-free DMEM/F-12 not containing ASC-CM. According to our preliminary studies results [13], we chose to evaluate fibroblasts migration at 24 h (the migration of fibroblasts was most active at this time point after being stimulated by 50% ASC-CM). The migrated fibroblasts were digested by trypsin-EDTA and counted under microscopy. After that, to compare the effects of ASC-CM and each cytokine, another experiment group was designed: the culture medium in the lower chamber was changed with DMEM/F12 with EGF, PDGF-AA, VEGF, or bFGF (at their optimal concentration). The above result of 50% ASC-CM was quoted and the assay procedure was the same as mentioned previously. All experiments were done in triplicate.

In scrape-wound healing assay, fibroblasts were seeded into 12-well plates with culture medium until they reached 80% confluence. These monolayers were then scored with a sterile pipette tip to leave a plus shape scratch of approximately 0.4-0.5 mm in width. Culture medium was then immediately removed and changed with (i) 50% ASC-CM, or (ii) 50% ASC-CM with the optimal concentration of each cytokine, or (iii) 50% ASC-CM with the neutralizing antibody of each cytokine.

### 2.5. Proliferation Assays

The effects of the ASC-CM cytokines on fibroblasts proliferation were determined utilizing CCK-8 assay. Briefly, 2 × 10^3^ fibroblasts were seeded into the 96-well plates for 24 h to adhere. Then the medium was changed with (i) 50% ASC-CM with different concentrations of cytokines (EGF, PDGF-AA, VEGF, and bFGF at 0, 1, 10, 20, 50, and 100 ng/mL, resp.), (ii) 50% ASC-CM with the neutralizing antibody of each cytokine, or (iii) serum-free DMEM/F-12 not containing ASC-CM. After that, in order to compare the effects of ASC-CM and each cytokine, another experiment group was designed: the culture medium was also changed with DMEM/F12 with EGF, PDGF-AA, VEGF or bFGF (at their optimal concentration). The above result of 50% ASC-CM was quoted. We chose to evaluate the cell proliferation in its logarithmic growth phase (day 3). All experiments were performed five times.

### 2.6. Statistical Analysis

All values are expressed as the mean ± SD. Comparisons between the two groups were analyzed by Student *t*-test and among more than two groups by ANOVA and then followed by posthoc Fisher's LSD. A *P* value of <0.05 was considered significant. All analyses were performed with SPSS 16.0.

## 3. Results

### 3.1. Morphologies, Flow Cytometry, and Multidifferentiation

Primary fibroblasts were spindle-shaped and distributed in a radial or swirl configuration (Figure 1(a)), and nearly all of the cultural cells were positive for vimentin (Figure 1(b)) and negative for cytokeratin 15 (Figure 1(c)). Primary ASCs demonstrated polygonal or round morphology in 24 hours, then displayed similar fibroblast-like or spindle-shaped morphology around 2 days, and were distributed in clusters. In the analysis by flow cytometry, P3-P4 ASCs were positive for the surface markers CD13, CD44, CD90, and CD105 (>90% of the population) and were negative for CD14 and CD34 (Figure 1(d)). We could observe a significant number of intracellular lipid droplets stained with Oil-Red-O when ASCs were cultured in adipogenesis medium for 21 days (Figure 1(e)) and calcium deposits were present when ASCs were cultured under osteogenic conditions for 21 days, as shown by alizarin red staining (Figure 1(f)). The relative genes expression showed a clear trend, gradually increasing during the differentiation process (Figures 1(g) and 1(h)).

### 3.2. Protein Microarray Analysis of ASC-CM

ASC-CM was assayed to determine the cytokines secreted by ASCs. Microarray analysis showed that ASC-CM contained a variety of cytokines [14], and a total of 268 cytokines had a signal that exceeded that of the background by 300-fold after being normalized against the internal control (IC) (Table 1). In these cytokines secreted by ASCs, EGF (relative concentration is 396 ± 29.5), PDGF-AA (relative concentration is 363.5 ± 34.5), VEGF (relative concentration is 360.5 ± 64.5), and bFGF (relative concentration is 389.5 ± 76) had high expression in ASC-CM (Figures 2(a) and 2(b)), and according to the previous literatures, they might have significant effects on cell migration and proliferation.

### 3.3. Migration Assay of Fibroblasts in the Stimulation of 50% ASC-CM with Different Concentrations of Cytokines and Their Neutralizing Antibodies

To further characterize the effects of the various cytokines in ASC-CM on fibroblasts migration and to determine the most effective cytokines concentration, the responses of fibroblasts to 50% ASC-CM with different concentrations of various cytokines (EGF, PDGF-AA, VEGF and bFGF at 0, 1, 10, 20, 50, and 100 ng/mL, resp.) and their neutralizing antibodies were examined by transwell assay. Each group was compared with 50% ASC-CM group without any additional cytokines. The results shown in Figure 3 indicated that bFGF, VEGF, and PDGF-AA promoted migration of fibroblasts, and their promoting effects were inhibited significantly by neutralizing antibodies (*P* < 0.05), while EGF had no significant promoting effect on fibroblasts migration. Figure 3 also indicated that the optimal concentrations of bFGF and VEGF were both 20 ng/mL (*P* < 0.01), while that of PDGF-AA was 50 ng/mL (*P* < 0.05). Furthermore, the promoting effect of 50% ASC-CM on fibroblasts migration was more significant than that of the control group (not containing ASC-CM) and each single cytokine group, specially more significant than the effect of EGF (*P* < 0.01) (Figure 3(a)). Simultaneously, the effects on fibroblasts migration were also further confirmed by scrape-wound healing assay (Figure 5).

### 3.4. Proliferation Assay of Fibroblasts in the Stimulation of 50% ASC-CM with Different Concentrations of Cytokines and Their Neutralizing Antibodies

To further characterize the effects of the cytokines in ASC-CM on fibroblasts proliferation and to determine the optimal cytokine concentration, we examined the responses of fibroblasts to 50% ASC-CM with different concentrations of the cytokines (EGF, PDGF-AA, VEGF, and bFGF at 0, 1, 10, 20, 50, and 100 ng/mL, resp.) and their neutralizing antibodies. The results at day 3 were chosen to compare the effects of these cytokine at the respective concentrations, as day 3 was a time point of the logarithmic growth phase during which the cells proliferated significantly. The results shown in Figure 4 indicated that EGF and bFGF promoted fibroblasts proliferation, and their effects were significantly inhibited by neutralizing antibodies (*P* < 0.05), while PDGF-AA and VEGF had no significant promoting effect on fibroblasts proliferation. Figure 4 also indicated that the optimal concentration of EGF was 50 ng/mL (*P* < 0.05), and that of bFGF was 20 ng/mL (*P* < 0.05) (there were no significant differences among 20 ng/mL bFGF, 50 ng·mL bFGF, and 100 ng/mL bFGF groups). Furthermore, the promoting effect of 50% ASC-CM was more significant than that of the control group (not containing ASC-CM) and each single cytokine group.

## 4. Discussion

Dermal fibroblasts play a necessary role during the cutaneous wound healing [15, 16]. In the early stage of the wound healing, the proliferation and migration of dermal fibroblasts are activated, which are essential for wound contraction, extracellular matrix deposition, and tissue remodeling. In addition, wound repair is a complex process which depends on the interaction between the effector cells and cytokines, including EGF, PDGF-AA, VEGF, and bFGF [17]. ASCs have been demonstrated to have promoting effect on skin wound healing [18]. In our previous studies [13], we have also determined that the ASC-CM was of benefit to the migration and proliferation of fibroblasts, keratinocytes, and endothelial cells, and these phenomena implicated the effectiveness of paracrine mechanism of ASCs. However, there are no definite answers to the questions. (1) What kinds of cytokines are there in the ASC-CM? (2) Which cytokine in ASC-CM plays more important role in the migration and proliferation of the dermal fibroblasts? (3) Is the effect of ASC-CM on the wound healing better than of a single cytokine?

To answer the questions above, in the present study, ASC-CM protein microarray analysis was performed to determine the concentrations of EGF, PDGF-AA, VEGF, and bFGF, which were demonstrated with significant promoting effect on the migration and proliferation of functional cells in wound healing [19–22]. They all had a signal that exceeded 300-fold. The result suggested that the four kinds of cytokines may play important roles in the wound healing by the paracrine mechanism of ASCs.

Among the four kinds of cytokines above, EGF family may be the best-characterized growth factors in wound healing. A growing body of studies has demonstrated that EGF can accelerate reepithelialization by increasing the proliferation and cell migration of keratinocytes in acute wound [23–27]. V. Frelrd et al. [20] demonstrated the effect of EGF on fibroblasts proliferation, and our results confirmed the former result. In our study, EGF promoted the proliferation of fibroblasts. Along with the increase of EGF concentration, its promotional effect became progressively more powerful, and the plateau level of EGF appeared at concentration of 50 ng/mL, while this effect was significantly (*P* < 0.05) inhibited by its neutralizing antibody. However, there is limited understanding about the effect of EGF on migration. In the study, the detection result of migration was a little complicated when fibroblasts were stimulated by EGF. The migration of fibroblasts was (*P* < 0.01) promoted by EGF at a low concentration (1 ng/mL), but with the increase of concentration, the migrated cells number began to reduce, reaching the bottom at the concentration of 20 ng/mL, and then gradually picked up at the higher concentrations (>20 ng/mL), increasing most significantly at the concentration of 100 ng/mL (*P* < 0.05). A possible reason for this phenomenon is that EGF is a cytokine related to cell mitosis and exerts a significant effect on fibroblasts proliferation. Therefore, its effect on proliferation might obscure the effect on migration when it was at the higher concentrations of EGF (≥20 ng/mL).

A lot of evidence demonstrated the effect of bFGF, PDGF-AA, and VEGF on promoting the proliferation and migration of fibroblasts [28, 29]. In our study, bFGF promoted the proliferation of fibroblasts, and with the increase of bFGF concentration, its promotional effect became progressively more powerful; the plateau level of bFGF was at 20 ng/mL (no more significant promoting effect with higher concentration). This effect was significantly (*P* < 0.05) inhibited by its neutralizing antibody. In addition, bFGF, VEGF, and PDGF-AA promoted fibroblasts migration in such a manner that, as the concentration of cytokines increased, their effect became progressively more powerful and the plateau level of bFGF was at 20 ng/mL, VEGF at 20 ng/mL, and PDGF-AA at 50 ng/mL. Once again, this effect was significantly (*P* < 0.05) inhibited by their neutralizing antibodies. These results suggested that bFGF was the main cytokine in ASC-CM promoting not only the proliferation but also the migration of fibroblasts. However, VEGF and PDGF-AA in ASC-CM only had a significant promoting effect on fibroblasts migration, with no significant effect on fibroblasts proliferation.

ASCs have demonstrated the effect of promoting the skin wound healing [18]. There is also ample evidence based on studies *in vitro* and *in vivo* to demonstrate that ASC-CM has effect of promoting skin wound healing due to the growth factors, cytokines, and chemokines [7–9]. However, there is limited understanding about whether the effect of ASC-CM on the wound healing is better than single cytokine. In our study, our results shown in Figure 2 and Figure 3 suggested that either on the migration or the proliferation of fibroblasts, the effect of ASC-CM was better than EGF, PDGF-AA, VEGF, or bFGF. On the other hand, we determined that the signal of 57 cytokines in ASC-CM exceeded 300-fold. Some cytokines, such as angiopoietin-1, 4, endothelin, TSP, IL-22, and EDA-2, have already demonstrated the effect of promoting the cutaneous wound healing [30–35]. As a result, the effect of ASC-CM on the wound healing which was better than single cytokines may be explained partly.

## 5. Conclusion

In summary, ASC-CM promotes the proliferation and migration of skin fibroblasts, and a variety of bioactive factors in ASC-CM work together to promote wound healing. Therefore, compared to the individual application of commercially prepared cytokines, ASC-CM has better prospects for highly positive clinical applications. However, wound healing *in vivo* is a much more complex biological process, so more *in vivo* studies are needed on the effects of these cytokines on fibroblast proliferation and migration. In addition, the effects and mechanisms of other cytokines on wound healing will be investigated in the future studies.

## Figures and Tables

**Figure 1:** Isolation and identification of human fibroblasts and ASCs *in vitro*. Fibroblasts were spindle-shaped (a) and positive for immunofluorescence staining of vimentin (b), while negative for cytokeratin 15 (c). ASCs were identified by flow cytometry of mesenchymal stem cells markers (d) and multiple differentiations. Adipogenesis of ASCs was confirmed by Oil-Red-O staining (e) and gene expressions of PPAR-*γ* (g). Osteogenesis was confirmed by alizarin red staining (f) and gene expression of Runx2 (h).

**Figure 2:** Protein microarray analysis of ASC-CM (a) and relative concentrations of EGF, PDGF-AA, VEGF, and bFGF in ASC-CM (b).

**Figure 3:** The effects of different concentrations or the neutralizing antibodies of cytokines in the 50% ASC-CM or DMEM on skin fibroblasts migration utilizing transwell assay. Migration was observed to be inhibited by EGF at 20 ng/mL, while being obviously promoted at 100 ng/mL (a). Fibroblasts migration was significantly promoted by PDGF-AA at 50 ng/mL (the optimal concentration) and 100 ng/mL, and the promoting effect was obviously inhibited when neutralizing antibody of PDGF-AA was added (b). VEGF was observed to make contribution to fibroblasts migration, and the optimal concentration was 20 ng/mL (*P* < 0.01), while this contribution was restrained by its neutralizing antibody (*P* < 0.05) (c). The bFGF at 20 ng/mL (the optimal concentration), 50 ng/mL, and 100 ng/mL obviously promoted fibroblast migration (*P* < 0.05), and its neutralizing antibody obviously inhibited fibroblast migration (*P* < 0.05) (d). In addition, compared with the control group (not containing ASC-CM) and each single cytokine group, specially the EGF, 50% ASC-CM significantly promoted the fibroblasts migration. *(*P* < 0.05); **(*P* < 0.01); NA: neutralizing antibody group. Each group was compared with 50% ASC-CM without any additional cytokines.

**Figure 4:** The effects of 50% ASC-CM with different concentrations of cytokines on proliferation of skin fibroblasts. The proliferation of fibroblasts was obviously promoted by EGF at 50 and 100 ng/mL (a) and also by bFGF at 20, 50, and 100 ng/mL (b), and their promoting effects were both inhibited by their neutralizing antibodies. However, PDGF and VEGF might not significantly contribute to fibroblasts proliferation (c and d). In addition, the promoting effect of 50% ASC-CM on fibroblasts proliferation was more significant than that of the control group (not containing ASC-CM) and each single cytokine. *(*P* < 0.05); **(*P* < 0.01); NA: neutralizing antibody group.

**Figure 5:** The effects of EGF, VEGF, PDGF, and bFGF in 50% ASC-CM on skin fibroblasts migration utilizing scrape-wound healing assay, and the optimal concentration of cytokines (reference to the result of transwell assay) in 50% ASC-CM was chosen to further confirm its effect. Results showed that fibroblasts migration was exactly inhibited by 20 ng/mL of EGF (b, g), while it was promoted by 20 ng/mL VEGF (c, h), 50 ng/mL PDGF (d, i), and 20 ng/mL bFGF (e, j). Their effects could be restrained by their neutralizing antibody (k–n). This result was consistent with the transwell assay.

**Table 1:** Cytokines whose internal control normalizations without background exceeded 300 folds in ASC-CM.

Cytokine	Internal control
EDA-A2	10056 ± 198
IGFBP-rp1/IGFBP-7	6651 ± 101.5
Thrombospondin (TSP)	4544.5 ± 67.5
TIMP-1	3221.5 ± 43
SPARC	2607 ± 51
GDF3	1400.5 ± 42.5
NRG3	1328.5 ± 32
HCR/CRAM-A/B	1261 ± 28
MSP alpha chain	1253.5 ± 23.5
MMP-20	1085 ± 12.5
APRIL	895.5 ± 27.5
LIF R alpha	893.5 ± 54
TGF-beta 5	839 ± 43.5
IL-22	811.5 ± 21.5
FGF-11	800.5 ± 19.5
MMP-25/MT6-MMP	763.5 ± 21
IL-20 R alpha	752 ± 13.5
IL-1 F5/FIL1 delta	742 ± 45.5
CCR2	731 ± 12.5
IL-17D	715 ± 38
CNTF	704 ± 33
FGF R4	697 ± 100
Internal control	697 ± 34.5
SIGIRR	671.5 ± 46.5
IL-1 F9/IL-1 H1	655.5 ± 27.5
Hepassocin	639 ± 46.5
Lipocalin-1	639 ± 29
Luciferase	635.5 ± 20.5
Neurturin	633 ± 32
IL-20	632 ± 29.5
IL-29	632 ± 17.5
MIP-3 alpha	628 ± 19
Angiopoietin-like 1	627.5 ± 39.5
sFRP-3	622 ± 23.5
NT-3	616 ± 67.5
Lymphotoxin beta/TNFSF3	606.5 ± 34.5
IL-1 F6/FIL1 epsilon	602 ± 55
IL-17E	599 ± 49
MMP-10	596.5 ± 37
NRG1-beta 1/HRG1-beta 1	596 ± 20.5
Glypican 3	595.5 ± 29
IL-1 F7/FIL1 zeta	593 ± 23
IL-19	592 ± 23.5
TACI/TNFRSF13B	590 ± 14.5
IL-1 ra	583.5 ± 29.5
IL-17B R	575 ± 35
MMP-7	566.5 ± 29
Dkk-4	560 ± 40
IL-26	558.5 ± 46.5
M-CSF R	549 ± 28.5
Follistatin-like 1	547 ± 43
MIP-1b	542 ± 59
Insulin R	541 ± 34.5
Endothelin	540 ± 19.5
MIP-1a	540 ± 61
I-TAC/CXCL11	535 ± 25.5
RELT/TNFRSF19L	529.5 ± 38.5
CTGF/CCN2	524 ± 34.5
CCR4	523.5 ± 39
Endoglin/CD105	521 ± 61
EDG-1	515 ± 43
Activin C	510 ± 56.5
MMP-11/stromelysin-3	509.5 ± 37
CXCR2/IL-8 RB	503.5 ± 38.5
IL-1 R9	501 ± 32.5
MMP-1	501 ± 17.5
GDF5	498 ± 28
BMP-8	493 ± 45.5
Dkk-1	492 ± 21
IGF-II	486 ± 32
TMEFF1/tomoregulin-1	486 ± 29.5
IL-7 R alpha	482 ± 39.5
IL-15 R alpha	480.5 ± 32
Heregulin/NDF/GGF/neuregulin	478 ± 54.5
CCR9	477.5 ± 21
BMP-5	476.5 ± 93
Siglec-9	476.5 ± 85.5
IL-4 R	474 ± 39.5
CCR1	472.5 ± 21.5
OX40 ligand/TNFSF4	471.5 ± 39
VEGF R2 (KDR)	469.5 ± 38.5
MMP-15	467.5 ± 75.5
P-selectin	465.5 ± 25.5
G-CSF R/CD 114	464 ± 79.5
IL-24	462.5 ± 75
E-Selectin	461.5 ± 56
IL-5 R alpha	459 ± 25.5
L-Selectin (CD62L)	458.5 ± 19
HB-EGF	458 ± 11.5
Growth hormone (GH)	457.5 ± 26.5
IL-17F	456 ± 39.5
PF4/CXCL4	456 ± 91.5
MMP-3	455 ± 62
IL-17C	454 ± 39
Inhibin B	453.5 ± 38.5
Sonic hedgehog (Shh N-terminal)	453 ± 87.5
MDC	452.5 ± 34.5
Neuritin	451 ± 61.5
CCR5	450.5 ± 55
CXCR6	450.5 ± 61
IGF-I SR	449.5 ± 23.5
LIGHT/TNFSF14	446 ± 57.5
HGF	444 ± 34.5
Eotaxin-3/CCL26	443.5 ± 95.5
Erythropoietin	443.5 ± 88
GDNF	443.5 ± 62
TNF RII/TNFRSF1B	439.5 ± 57
Prolactin	438 ± 36.5
Adiponectin/Acrp30	436 ± 45.5
IL-12 p40	435 ± 93.5
CTLA-4/CD152	433.5 ± 67.5
BMPR-II	431.5 ± 41.5
LIF	431 ± 57.5
TECK/CCL25	430.5 ± 44.5
Pref-1	430 ± 32
IL-6 R	429 ± 79.5
IL-17B	429 ± 56.5
IL-12 p70	427 ± 48
DR6/TNFRSF21	426.5 ± 65.5
FGF-16	425 ± 42.5
IGFBP-6	424.5 ± 30.5
IL-17R	424 ± 92
Osteoprotegerin/TNFRSF11B	423 ± 21.5
Thrombospondin-2	421 ± 87.5
TREM-1	420 ± 67
Angiopoietin-like 2	419.5 ± 34.5
S100 A8/A9	418 ± 67.5
CXCR1/IL-8 RA	417 ± 54.5
LFA-1 alpha	417 ± 73
Dtk	416.5 ± 48.5
IL-12 R beta 1	416.5 ± 23
MMP-13	416.5 ± 37
SCF	414.5 ± 45.5
FGF-10/KGF-2	413 ± 82.5
NRG2	412 ± 11
B7-1/CD80	411.5 ± 32.5
FGF-9	410.5 ± 44
sgp130	408 ± 45.5
TIMP-2	408 ± 67.5
ALCAM	407.5 ± 32.5
GDF9	407 ± 37.5
HVEM/TNFRSF14	407 ± 34
BMP-4	405.5 ± 81.5
IL-1 sRI	403.5 ± 23.5
FGF R3	403 ± 22.5
AgRP	402.5 ± 32.5
TGF-beta 2	402.5 ± 92.5
SCF R/CD117	400.5 ± 11
SDF-1/CXCL12	400 ± 19
IL-22 BP	397 ± 32.5
EGF	396 ± 29.5
VEGF-D	395 ± 83.5
NOV/CCN3	394.5 ± 66
Fas ligand	393.5 ± 21
Activin RIA/ALK-2	393 ± 39.5
BMPR-IA/ALK-3	393 ± 33.5
CCR6	393 ± 29.5
IL-21 R	392.5 ± 21.5
M-CSF	391.5 ± 54
LRP-6	391 ± 34
FGF Basic	389.5 ± 76
CD40/TNFRSF5	388.5 ± 21.5
MIF	388.5 ± 43
GDF11	386 ± 36
D6	385 ± 29
IL-23 R	384 ± 18.5
CRIM 1	383.5 ± 63.5
FLRG	383.5 ± 44
GFR alpha-4	383 ± 39
IL-10 R alpha	383 ± 23
Leptin R	382.5 ± 49.5
IL-18 BPa	380 ± 49.5
IL-13 R alpha 1	379 ± 33
uPA	378.5 ± 17.5
CD40 ligand/TNFSF5/CD154	378 ± 21
IL-1 R6/IL-1 Rrp2	378 ± 32
TIMP-4	377.5 ± 19
CLC	377 ± 18.5
MCP-3	376.5 ± 21.5
OSM	375.5 ± 23
RANTES	375 ± 57
I-309	374 ± 46
TRAIL/TNFSF10	374 ± 33
MMP-8	371.5 ± 11.5
NT-4	371 ± 29.5
GDF-15	370 ± 21
CD27/TNFRSF7	369.5 ± 39.5
CXCL14/BRAK	368.5 ± 87
Follistatin	368.5 ± 34
CXCR5/BLR-1	367 ± 32.5
FGF-4	367 ± 29
MSP beta-chain	366.5 ± 39.5
RANK/TNFRSF11A	366.5 ± 82
Siglec-5/CD170	366 ± 71
Ubiquitin+1	365.5 ± 34.5
PDGF-AA	363.5 ± 31.5
DAN	363 ± 32
Tie-2	362.5 ± 45
Angiopoietin-like factor	361.5 ± 23
CCR7	361.5 ± 49.5
VEGF	360.5 ± 64.5
IL-18 R beta/AcPL	359 ± 17
MMP-2	359 ± 29.5
Tie-1	359 ± 11
BDNF	358.5 ± 32
HCC-4/CCL16	357 ± 37.5
Thrombopoietin (TPO)	357 ± 45.5
Thrombospondin-1	355.5 ± 67.5
IGFBP-3	355 ± 78.5
Vasorin	355 ± 27.5
Tarc	354.5 ± 98.5
IL-2 R beta/CD122	353 ± 43
Lymphotactin/XCL1	353 ± 66
Angiopoietin-1	352.5 ± 45
IGFBP-1	352.5 ± 18.5
Pentraxin 3/TSG-14	352 ± 21
GREMLIN	347 ± 43
GITR/TNFRF18	345 ± 43.5
CCR3	343 ± 55.5
Angiopoietin-4	342.5 ± 36.5
DcR3/TNFRSF6B	342.5 ± 11.5
CCR8	341.5 ± 23.5
TGF-beta RII	341.5 ± 19.5
Activin B	340.5 ± 22.5
CCL28/VIC	338.5 ± 61
ErbB4	338.5 ± 17.5
IFN-gamma R1	337.5 ± 65
IL-3 R alpha	337 ± 32
CCL14/HCC-1/HCC-3	335.5 ± 18
TNF RI/TNFRSF1A	335 ± 11.5
Amphiregulin (AR)	333.5 ± 29
WIF-1	333.5 ± 32
Decorin	333.00
IL-1 beta	333 ± 22
TRAIL R4/TNFRSF10D	332.5 ± 45.5
TIMP-3	330 ± 64
FGF-13 1B	328 ± 45.5
Cardiotrophin-1/CT-1	326.5 ± 33
FGF-6	326.5 ± 19.5
TGF-beta RIII	326 ± 21
FGF-7/KGF	325 ± 38.5
EG-VEGF/PK1	324.5 ± 18
IL-2 R alpha	324.5 ± 32.5
GFR alpha-3	323.5 ± 44
RAGE	323.5 ± 45
DR3/TNFRSF25	323 ± 38
Orexin B	322.5 ± 23
Leptin (OB)	321.5 ± 21
TGF-beta 3	320.5 ± 15.5
IFN-beta	320 ± 32.5
IGFBP-2	316.5 ± 38.5
IL-10 R beta	314 ± 45
PDGF-BB	312.5 ± 25.5
MMP-9	311 ± 21
Cryptic	310.5 ± 13.5
TRAIL R1/DR4/TNFRSF10A	310 ± 26.5
Axl	309.5 ± 16
CXCR3	309.5 ± 34.5
GCP-2/CXCL6	309.5 ± 67
TNF-beta	309 ± 21
FGF-BP	308 ± 34
PD-ECGF	307 ± 26.5
sFRP-4	306 ± 17
uPAR	305 ± 23.5
Eotaxin/CCL11	303 ± 21
GRO	303 ± 13.5
MIG	301.5 ± 23
PARC/CCL18	300 ± 25.5
